# A Retrospective Analysis on the Effects and Complications of Endoscope-Assisted Transoral Approach and Lateral Cervical Approach in the Resection of Parapharyngeal Space Tumors

**DOI:** 10.1155/2022/7536330

**Published:** 2022-09-23

**Authors:** Danni Guo, Changling Sun, Xiao Yin, Hongyang Qu, Bingyi Dai, Lin Hu, Chen Zhou, Xiaodong Du

**Affiliations:** Department of Otorhinolaryngology-Head & Neck Surgery, Affiliated Hospital of Jiangnan University, Wuxi 214122, China

## Abstract

**Objective:**

To observe and compare the effects and complications of endoscope-assisted transoral approach and lateral cervical approach in the resection of parapharyngeal space (PSS) tumors.

**Methods:**

From January 2013 to September 2021, 69 patients with parapharyngeal space tumors in the Affiliated Hospital of Jiangnan University were divided into the control group (*n* = 37) and the observation group (*n* = 32) according to the mode of operation. The tumors in the parapharyngeal space were resected by the lateral cervical approach in the control group, and the tumors in the parapharyngeal space were removed by endoscopy-assisted transoral approach in the observation group. The general clinical data and operation conditions of the two groups, including operative blood loss, operation time, drainage volume and drainage time, hospital stay, perioperative pain degree, and tumor resection rate were collected and analyzed statistically. The patients were followed up for 6 months, and the complications of the two groups were recorded.

**Results:**

Compared with the control group, the operation time in the observation group was significantly shorter, and the amount of intraoperative bleeding in the observation group was significantly less than that in the control group, and the difference was statistically significant (*P* < 0.05). The postoperative drainage was less and the hospital stay in the observation group was shorter than that in the control group, and the difference was statistically significant (*P* < 0.05). There was no significant difference in tumor resection rate between the two groups. The visual analog scale (VAS) score on the 1st and 3rd day after operation in the observation group was lower than that in the control group. After treatment, some patients in the two groups had complications such as nerve injury, dysphagia, difficulty in mouth opening, massive hemorrhage, and parotid fistula. The total incidence of complications in the observation group was lower than that in the control group, and the difference was statistically significant (*P* < 0.05).

**Conclusions:**

The effect of the endoscope-assisted transoral approach is similar to that of the lateral cervical approach in the resection of tumors in parapharyngeal space, but the endoscope-assisted transoral approach has shorter operation time, less intraoperative bleeding, and less postoperative drainage. The indwelling time and hospital stay of the drainage device were shorter than those of the patients with transcervical approach, and the perioperative stress response of patients with endoscope-assisted transoral approach is mild, which is beneficial to the physical and mental recovery of the patients.

## 1. Introduction

Parapharyngeal space (PSS) tumors account for about 0.5% of head and neck tumors and generally occur in adults, 30–50 years old account for about 50%, occur in childhood is very rare, female incidence is more than male [1]. There are many kinds of tumors in PSS, with more than 70 kinds, but benign tumors account for 70–80%, malignant tumors account for 20–30%, including primary tumors, direct spread tumors, and distant metastatic tumors. It is recognized that the more common PSS tumors are pleomorphic adenoma, schwannoma, and paraganglioma [2, 3]. Considering the concealment of PSS, it is often difficult to detect PSS tumors in the early stage. It is generally believed that PSS tumor volume larger than 2.5 cm will lead to clinical symptoms, such as upper neck mass, lateral pharyngeal wall or glossopalatine arch surface eminence, throat foreign body sensation, sore throat, cough, dysphagia, tinnitus, snoring, and even dyspnea [4]. With the growth of the tumor, it will also lead to corresponding neurological dysfunction, characterized by hoarseness, ambiguous speech, limited mouth opening, Horner syndrome, and so on, which seriously affect the life of the patients [4]. The diagnosis of PSS tumors needs imaging examination for preoperative evaluation, according to the typical imaging features of the tumor to make a higher accuracy of preoperative diagnosis. The clinical diagnosis has a high coincidence rate. Ultrasound and CT-guided fine biopsy can make a preliminary judgment of the tumor before open operation and choose the appropriate mode of operation [5].

With regard to PSS tumors, complete surgical resection is the optimal choice for the therapeutic strategy [6]. Due to the diversity of tumor types and the complexity of anatomical structure in PSS, it is very important to choose a reasonable surgical approach in order to avoid neurovascular damage and even functional disorders [6]. In the continuous exploration of many clinicians and scholars, there are more surgical approaches, including lateral cervical incision, cervicomandibular approach, transcervical-parotid approach, transcaliber approach, and so on. In recent years, with the gradual development of endoscopic technology, clinicians have also investigated the feasibility of endoscopic-assisted transcaliber approach in the treatment of PSS tumors [7, 8]. With the further research of technology, endoscope-assisted minimally invasive surgery can remove many large and deep tumors in PSS. However, all kinds of surgical approaches have their advantages and disadvantages. According to the application experience of clinicians at present, it is acknowledged that the external cervical approach can fully expose the surgical field, and the important blood vessels and nerves can be protected to a certain extent, but due to the large scope of the operation and great trauma to the tissue, such as removal of the submandibular gland and amputation of the mandible in part of the operation, there are many postoperative complications, and there are scars on the face, influencing the appearance [9]. The trauma of the transcaliber approach is less than that of the external cervical approach, and there is no scar on the face, but due to the lack of surgical field, it has a certain blindness in separating the tumor and its surrounding tissue, and the scope of application is relatively limited. Traditionally, it is considered to be only suitable for relatively small tumors near the pharyngeal cavity [10]. Endoscope-assisted transoral minimally invasive treatment of PSS tumors avoid mandibular amputation, important neurovascular injury, and facial scar [11]. However, there are few clinical comparative studies on cervical incision and endoscope-assisted transcaliber approach in the treatment of PSS tumors. In order to provide references and suggestions for the selection of surgical approaches for PSS tumors, this study selected the complete clinical data of patients with PSS tumors and established relevant inclusion and exclusion criteria to exclude other interference factors other than the influence of surgery, so as to make the comparison more reasonable. Based on the above, the purpose of this article was to observe and compare the efficacy and complications of endoscopic-assisted transoral and lateral cervical approaches in parapharyngeal space (PSS) tumor resection.

## 2. Patients and Methods

### 2.1. Clinical Information

From January 2013 to September 2021, 69 patients with parapharyngeal space tumors in the Affiliated Hospital of Jiangnan University were divided into the control group (*n* = 37) and the observation group (*n* = 32). All patients were diagnosed based on imaging manifestations and pathological findings. There were 18 males and 19 females in the control group. The patients in the control group ranged in age from 15 to 76 years, and the average age was (48.05± 15.62) years. Their course of disease ranged from 2 months to 36 months with an average of (12.11 ± 9.27) months. In the observation group, there were 14 males and 18 females. The patients in the observation ranged in age from 22 to 73 years, and the average age was (51.78 ± 13.89) years. The course of disease ranged from 1 months to 24 months with an average of (10.06 ± 6.54) months. The main clinical symptoms of the patients were neck swelling and pain, sleep snoring, hoarseness, foreign body sensation in the throat, dysphagia, inarticulate speech, tinnitus, and tightness, and even some cases had symptoms of holding breath and dyspnea in the lateral position, and a few patients had no obvious clinical symptoms. A mass was found inadvertently or during physical examination. Main signs: upper neck or submandibular mass; soft palate eminence of gloss palatine arch; protuberance of lateral wall of pharynx; and all patients underwent double diagnostic examination of oral cavity and neck. Auxiliary examinations included neck CT and/or MRI, polysomnography, and esophageal barium meal radiography, all of which were diagnosed as parapharyngeal space tumors before operation. Inclusion criteria (1) patients with parapharyngeal space tumors were diagnosed by cervical CT and/or MRI, polysomnography, esophageal barium meal radiography, and pathological examination; (2) it accords with the indication of surgical treatment; and (3) the patients and their families informed consent and signed the informed consent form. Exclusion criteria: (1) patients with other neurological diseases, nasopharynx, oral, esophageal tumors, and cognitive impairment that may lead to difficulty in mouth opening; (2) patients with severe malnutrition, malignant tumors, systemic immune system diseases, or major organ dysfunction and elderly patients; (3) patients with severe heart, kidney, liver, and other important organ dysfunction; and (4) do not want to participate in this study.

### 2.2. Treatment Method

The tumors in the parapharyngeal space were resected by the lateral cervical approach in the control group, and the tumors in the PSS were resected by endoscope-assisted transoral approach in the observation group.

Lateral cervical approach: behind the cervicomaxillary angle, from the top of the mastoid, down along the anterior edge of the sternocleidomastoid muscle to the level of the great angle of the hyoid, cut open the skin and subcutaneous tissue. Lifted the platysma myocutaneous flap, exposed the inferior pole of the parotid gland and the submandibular gland, pulled the sternocleidomastoid muscle backward, exposed the posterior abdomen of the digastric muscle, carefully dissected the internal carotid artery, external carotid artery, internal jugular vein, and vagus nerve; dissected the marginal branch of the facial nerve at the inferior margin of the mandible and the facial artery; separated the ancient inferior nerve from the deep surface of the digastric muscle; and dissected and protected the accessory nerve at 1/3 on the posterior edge of the sternocleidomastoid muscle. The tumor could be fully exposed by cutting off the styloid hyoid muscle and the posterior abdomen of the digastric muscle. If the tumor was located in the upper part of the PSS near the skull base, part of the mandibular angle bone should be removed (generally, the width of the resection area should not exceed 1/2 of the width of the mandible and the length should not exceed 3 cm) to expose the tumor completely. If it is close to the tumor capsule and separated carefully, the tumor can be removed sharply. After resection, the operative cavity was washed with iodophor and normal saline, negative pressure drainage was placed, and the incision was sutured layer by layer. The drainage tube stayed for two to three days. This surgical method is suitable for the resection of most PSS tumors, including some limited malignant tumors.

The operation of endoscope-assisted transoral approach: before operation, patients were treated with shoulder pads in supine position, head tilted back, and Davis mouth opener was placed through mouth to expose oropharynx. The front end of the red children's catheter was placed into the bottom of the nose through the anterior nostril, reaching back to the posterior nostril to the nasopharynx, down to the mouth, pulling the catheter out of the mouth, knotting and fixing both ends of the catheter at the upper lip, so as to pulled the soft palate forward to better expose the field of operation. Under nasal endoscope, at the tonsillar fossa of the lateral wall of the pharynx, a low-temperature plasma scalpel (Arthrocare Corporation EIC 5874-01, USA) was used to make a longitudinal incision from top to bottom. Incision of mucous membrane and submucous tissue (if the tonsil was too large and affected the visual field of operation, tonsillectomy should be performed first), exposed the superior constrictor of pharynx, dissected and separated the superior constrictor of pharynx, reached the surface of the tumor, closed to the tumor and separated the tumor capsule with plasma scalpel (COBLATE Level 7), the separation sequence should be paid attention to (see Figure 1). In order to avoid damaging the important blood vessels and nerves around the tumor due to blocking the visual field, we started from the inner side of the tumor, then turned to the front of the tumor, then separated the upper and lower parts of the tumor, and finally separated the outer side and back of the tumor. The separation should be gentle, avoid violence, and be carefully separated along the gap between the tumor capsule and the surrounding tissue. If adhesion between the capsule and surrounding tissue is found during separation, carefully separate it with vascular forceps, cut it open with a plasma scalpel under endoscope, and be operated by two surgeons. If necessary, the assistant could hold the endoscope, and the operator could operate with both hands. During the operation, the assistant held the suction device to suck the field bleeding in time to ensure the clarity of the operation field under the microscope (see Figure 2). If the amount of bleeding was more, you could use gauze to stop the bleeding first, and after the tumor was completely removed, carefully looked for the bleeding point and stopped the bleeding with plasma scalpel (COAG Level 3). If the size of the tumor was too large to be completely removed, the tumor could also be removed step by step. After tumor removal, we carefully checked whether there was bleeding in the operative cavity, rinsed the operative cavity alternately with iodophor and normal saline, and sutured the muscle and the mucous membrane of the pharyngeal wall layer by layer. The iodoform gauze was placed in the operative cavity according to the intraoperative conditions to drain the exudate from the operative cavity, stayed for two to three days. After operation, cephalosporins and tinidazole were given intravenously to prevent infection and, if necessary, corticosteroids were used intravenously to reduce edema in the operative area.

Surgical instruments and equipment: endoscopy and monitoring using KarlStorz company of Germany nasal endoscope products (0°mirror, diameter 4.0 mm, video surveillance system); low-temperature plasma scalpel (Arthrocare Corporation EIC 5874-01, USA); ultrasonic knife (Johnson Company HAR9F, USA); unipolar needle electric knife; and conventional surgical instruments.

### 2.3. Observation Index

(1) Operating time, (2) the amount of intraoperative bleeding, (3) postoperative drainage and drainage time, (4) instruct the patient to spit out oral secretions to estimate the amount of bleeding, (5) the amount of fluid and bleeding in the external cervical drainage tube, (6) the time from operation to discharge, and (7) visual analog score (VAS) was used to evaluate the pain degree of perioperative patients [12]. Using the 10 cm swimming scale, the 0 end indicates no pain, the 10 end indicates the most severe pain, and the score range is 0–10 points. The higher the score, the more severe the pain (8) tumor resection rate and (9) complications occurred within 6 months after operation.

### 2.4. Statistical Analysis

SPSS 23.0 statistical software was adopted to process the data. The measurement data were presented as ($\bar{x}\pm s$). The group design *t*-test was adopted for the comparison, and the analysis of variance was adopted for the comparison between multiple groups. Dunnett's *t*-test was adopted for comparison with the control group. The counting data were presented in the number of cases and the percentage. *χ*^2^ test was adopted for comparison between groups, and bilateral test was employed for all statistical tests.

## 3. Results

### 3.1. Comparison of Postoperative Pathological Results between the Two Groups

The pathological results showed that among the 32 patients in the observation group, there were 8 cases (25.00%) of nerve schwannoma, 6 cases (18.75%) of pleomorphic adenoma, 4 cases (12.50%) of branchial cleft cyst, 4 cases (12.50%) of elongated styloid process, 2 cases (6.25%) of hemangioma, 1 case (3.13%) of Warthin tumor, 1 case (3.13%) of paraganglioma, 5 cases (15.63%) of squamous cell carcinoma, and 1 case (3.13%) of synovial sarcoma; among the 37 patients in the control group, there were 13 cases (35.14%) of nerve schwannoma, 10 cases (27.03%) of branchial cleft cyst, 5 cases (13.51%) of pleomorphic adenoma, 2 cases (5.41%) of lipoma, 1 cases (2.70%) of hemangioma, 1 case (2.70%) of Warthin tumor, 1 case (2.70%) of paraganglioma, 1 case (2.70%) of lymphangioma, 1 cases (2.70%) of squamous cell carcinoma, 1 case (2.70%) of adenocarcinoma, and 1 case (2.70%) of pleomorphic liposarcoma.

The minimum diameter of the tumor in the observation group was 1.0 cm, the maximum diameter was 9.8 cm, and the average diameter was (3.86 ± 1.19) cm . In the control group, the minimum diameter was 1.2 cm, the maximum diameter was 8.0 cm, and the average diameter was (4.25 ± 1.37) cm. There was no significant difference in the above-mentioned indexes between the two groups (*P* > 0.05).

### 3.2. The Time of Operation and the Amount of Intraoperative Blood Loss between the Two Groups

Compared with the control group, the operation time of the observation group was significantly shorter and the amount of intraoperative blood loss was significantly less than that of the control group (*P* < 0.05). The results are shown in Table 1.

### 3.3. Comparison of Postoperative Drainage and Hospital Stay

Compared with the control group, the posterior drainage in the observation group was less, and the hospitalization time in the observation group was shorter than that in the control group, and the difference was statistically significant (*P* < 0.05). The results are shown in Table 2.

### 3.4. Comparison of Tumor Resection and Perioperative Pain

There was no significant difference in tumor resection rate between the two groups. The VAS score of the observation group was lower than that of the control group at 1st day and 3rd day after operation, and the difference was statistically significant (*P* < 0.05). The results are shown in Table 3.

### 3.5. The Incidence of Complications after Surgical Treatment between the Two Groups

After treatment, complications such as nerve injury, dysphagia, difficulty in mouth opening, massive hemorrhage, and parotid fistula occurred in both groups. The total incidence of complications in the observation group was significantly lower than that in the control group, and the difference was statistically significant (*P* < 0.05). The results are shown in Table 4.

## 4. Discussion

The position of the PSS is deep, from the base of the skull to the hyoid plane, which is the potential space of the head and neck with complex anatomical relationship [12]. PSS tumors are relatively rare, accounting for about 0.5% of head and neck tumors, including benign tumors (80%) and malignant tumors (20%). The most common is pleomorphic adenoma originating from the parotid gland, followed by neurogenic tumors (including schwannoma, neurofibroma, and paraganglioma) [13]. The early clinical symptoms of PSS tumor are not obvious and are easy to be ignored. Because of its deep location, most patients will be inadvertently found during a health examination. When the diameter of PSS tumor is larger than 3 cm, pharyngeal mass, neck mass, pain, foreign body sensation, dysphagia, and even dysphagia may occur due to tumor invasion of pharyngeal cavity or adjacent tissues [14]. Horner syndrome, which occurs when sympathetic nerves are compressed, is typically characterized by myosis, ptosis, and decreased sweat. Local expansion of the tumor can compress the sympathetic nerve, causing snoring, dyspnea, and other compression symptoms [15, 16]. The previous study unveiled that most patients had no obvious characteristic clinical manifestations, especially in the early stage of the disease. About 36% of the patients had ear tightness and earache, 13% of the patients had dysphagia, 11% of the patients had hearing loss, 10.5% of the patients had hoarseness, and about 6.4% of the patients had facial and lower jaw pain [17], suggesting that clinicians should carefully inquire the medical history of atypical clinical symptoms and make detailed examinations when receiving such patients, so as to avoid misdiagnosis and mistreatment.

Therefore, preoperative examination and evaluation is particularly indispensable for the therapeutics of PSS tumors. The more intuitive method in the diagnosis and examination of tumors in the PSS is to first use the method of joint diagnosis with both hands to understand the size, texture, location, and range of activity of the tumor, such as carotid body tumor can touch the sense of pulsation and have a certain degree of compression, therefore, the tumor can move in the anterior and posterior position but not up and down [18]. However, because of the deep location of PSS, it is difficult to accurately estimate the size of the tumor and its relationship with the surrounding tissue and important structures, so imaging examination is particularly important for the preoperative evaluation of PSS tumors. Through CT or MRI examination, we can understand the degree of tumor involvement and its relationship with the surrounding important tissues, such as the relationship with carotid sheath, skull base, and intracranial invasion, so as to help clinicians to judge in time and determine the operation plan [19, 20].

Surgical treatment still remains the optimal choice for PSS tumors [21]. Due to the various pathological types, deep anatomical location and complex surrounding structure of tumors in the PSS, the selection of appropriate surgical approach is the key to successful operation. In order to formulate the surgical approach before operation, we should focus on the size and nature of the tumor and its relationship with the surrounding important blood vessels and nerves and choose a surgical approach that can fully expose the operative field and remove the tumor completely. Meanwhile, it is the principle of surgical treatment of PSS tumors that can avoid damage to important blood vessels and nerves and minimize postoperative scars and deformities.

Low-temperature plasma (LTP) technology has emerged in recent years, and its application in the neck has proven to be successful such as tonsillectomy and adenoidectomy. The low-temperature plasma scalpel is composed of a conductive medium (sodium) that generates a high concentration of plasma around the electrode, which is made up of highly ionized particles. Because the current does not generate a large amount of heat through the tissue and does not cause visual damage to the tissue, such particles have quite enough energy to detach the molecular bonds in the material, which in turn differs various molecules and reduces the tissue. At the same time, the characteristics of ultralow temperature and strong hemostatic effect of plasma can completely cut off the tumor tissue. Low-temperature plasma scalpel also has some disadvantages. First of all, it is difficult to decompose the levels and anatomical structures of some tissues during the operation, which will lead to tissue damage. Second, the temperature parameters during the operation are not easy to control, which may lead to vascular injury and tissue perforation, resulting in a series of complications. The incision is tiny and the ablation depth can be carefully regulated due to the extremely low working temperature, causing less injury to the surrounding skin during the procedure.

Transcervical approach is the most commonly used surgical approach for PSS tumors [22]. It is suitable for most patients with PSS tumors, with these advantages: (1) large operating space, directly entering the PSS, better exposing the important blood vessels and nerves in the PSS, and can avoid the injury of parotid gland and facial nerve; (2) can better protect the internal and external carotid arteries; (3) it is easy to separate the blood vessels at the edge of the tumor, and it is convenient to stop bleeding. However, the transcervical approach will bring greater surgical trauma to the patients, and the postoperative incision scar is larger, which will bring psychological burden to the patients. In addition, in order to completely remove the tumor during the operation, it is necessary to cut off part of the nerves and blood vessels, increasing the risk of facial nerve injury. Some scholars believe that the lateral cervical approach is limited in the treatment of tumors and angiogenic tumors located in the medial or upper part of PSS [22].

The resection of tumors in PSS by transoral approach was first proposed by Goodwin and Chandler [23]. The advantages of this approach are direct surgical approach, simple operation, less surgical trauma, early oral feeding, no surgical scar in the neck, and shorter hospitalization time [24]. However, in the past, since the surgical approach was operated in the oral cavity, restricted by lighting equipment and other surgical instruments, the operative field was narrow, it was difficult to expose during the operation, and it was blind to separate the tumor during the operation. Moreover, it is prone to bring about important vascular and nerve injury in the PSS, parotid gland leakage in the PSS, and incomplete tumor resection and other adverse consequences [24]. Some scholars believe that the transoral approach is only suitable for benign nonvascular PSS tumors whose diameter in the anterior styloid space is less than 3 cm, especially those with intact capsule protruding to the oropharynx [24]. However, the operative complications and postoperative discomfort induced by transcervical, transparotid and transmandibular approach were significantly more than those induces by transoral approach [25, 26]. In recent years, with the development of endoscopic technology, since the application of endoscopic technology in clinical surgery has the advantages of good lighting, clear surgical field and wide visual angle, it is possible to remove deep tumors through natural spaces such as nasal cavity and oral cavity as much as possible. Endoscope-assisted transoral approach has been widely used, and it has been paid more and more attention by colleagues [27]. We believe that, considering that most PSS tumors are benign, among the many surgical methods of PSS tumor resection, only endoscope-assisted transoral approach can satisfy the complete resection of the tumor. At the same time, the principle of surgical treatment is to retain important vascular and neurological functions and minimize postoperative scars and deformities. Endoscope-assisted transoral approach not only has the advantages of traditional transoral approach but also solves the shortcomings of narrow visual field and difficult exposure [27].

In this study, there was no significant difference in the complete resection rate and residual rate of tumors in the PSS between the two groups (*P* > 0.05), indicating that the two surgical approaches can effectively remove tumors in the PSS, and the curative effect is the same. However, compared with the transcervical approach, the endoscope-assisted transoral approach had shorter operation time and less intraoperative bleeding, the postoperative drainage volume, indwelling time of drainage device, and hospital stay were less than those of transcervical approach, and the difference was statistically significant (*P* < 0.05). In a meanwhile, the VAS score of endoscope-assisted transoral approach was significantly lower than that of transcervical approach at 1st day and 3rd day after operation. In addition, the endoscope-assisted transoral approach can enlarge the surgical area several times, observe the lesions and microvessels that are easy to be ignored by the naked eye, and better remove the diseased tissue. Moreover, the use of low-temperature plasma equipment, cleaning, suction, electrocoagulation, and cutting into one can effectively reduce bleeding and shorten the time of operation. In contrast, the transcervical approach has a wide field of vision. Double-click electrocoagulation and meridian attractor are used during the operation, which need to cut open the skin, subcutaneous tissue and platysma muscle in turn, and suture after operation. Therefore, endoscope-assisted transoral approach surgery requires shorter time and less trauma, so intraoperative bleeding, drainage device indwelling time, hospital stay are less, and the degree of perioperative pain is relatively mild. However, no matter what kind of operation, psychological factors such as treatment operation and worrying about the consequences of treatment will cause patients' fear and anxiety and induce stress reaction to a certain extent. The stress reaction will lead to accelerated breathing, elevated blood pressure, and a series of changes in hormone levels, which is not conducive to the recovery of patients [27]. The stress response induced by endoscope-assisted transoral approach surgery is mild, which may be due to the shorter operation time and less trauma of the patients. After treatment, some patients in the two groups had complications such as nerve injury (hoarseness, facial paralysis, and weakness of shoulder lifting), dysphagia, mouth opening, massive hemorrhage, and parotid fistula. The total incidence of complications in the observation group was lower than that in the control group, and the difference was statistically significant (*P* < 0.05). Postoperative hoarseness occurred in 3 cases, which was related to cranial nerve injury in the posterior group, but hoarseness recovered within half a year after operation. 1 case with dysphagia had postoperative pain VAS score as high as 7, no pharyngeal edema and dyspnea occurred after operation, and the symptoms were alleviated within 10 days after operation. 3 cases with dysphagia and difficulty in opening mouth considered postoperative infection and cellulitis in parapharyngeal space, and the symptoms improved within a week after treatment with antibiotics and corticosteroids. 2 cases of massive hemorrhage were primary bleeding within 24 hours after operation, and external carotid artery DSA was performed to stop the bleeding. After operation, 2 cases of parotid fistula were caused by parotidectomy of deep lobe of parotid gland. The use of oral prosthetic membrane during the parotid approach surgery can effectively prevent the occurrence of postoperative salivary gland fistula. 4 cases of facial paralysis were considered as injury of marginal mandibular branch of facial nerve, but did not cause fracture and recovered one month after operation, and 1 case of weakness of shoulder lifting was considered as brachial plexus injury after operation. In the comparison of postoperative complications, the total incidence of complications in the transcervical approach group was higher than that in the transoral approach group. It shows that the risk of complications of endoscope-assisted transoral approach is lower than that of transcervical approach. In addition, there is no scar in the neck after the transoral approach, which plays a great role in promoting the physical and mental recovery of the patients. This study has some limitations: the sample size of this study is small, it belongs to a single-center study, and there is a certain deviation. There are patients' own factors and other confounding factors that may interfere with the accuracy of this study. In future research, we will carry out multicenter, large sample prospective studies, or we can draw more valuable conclusions.

To sum up, endoscope-assisted transoral approach is similar to lateral cervical approach in the resection of PSS tumors. But the endoscope-assisted transoral approach has less operation time, less intraoperative blood loss, and postoperative drainage. The indwelling time of the drainage device and the length of hospital stay of the patients treated by endoscope-assisted transoral approach are also shorter. In addition, the degree of perioperative pain and stress reaction of the patients undergoing endoscope-assisted transoral approach are mild, which is beneficial to the physical and mental recovery of the patients with PSS tumors.

## Figures and Tables

**Figure 1:** Surgical field of direct view in the endoscope-assisted transoral approach.

**Figure 2:** Surgical field of endoscopy in the endoscope-assisted transoral approach.

**Table 1:** Comparison of operation time and intraoperative blood loss ($\bar{x}\pm s$).

Group	*N*	Operation time (min)	Intraoperative bleeding volume (ml)
Control group	37	109.86 ± 33.95	162.43 ± 93.70
Observation group	32	91.72 ± 31.24	118.13 ± 78.46
*t*		2.296	2.110
*P*		0.025	0.039

**Table 2:** comparison of postoperative drainage and hospital stay ($\bar{x}\pm s$).

Group	*N*	Drainage volume (mL)	Hospitalization time (d)
Control group	37	24.05 ± 6.91	6.38 ± 1.54
Observation group	32	15.78 ± 6.43	5.50 ± 1.28
*t*		5.119	2.557
*P*		<0.01	0.013

**Table 3:** comparison of tumor resection and perioperative pain [*n* (%), $\bar{x}\pm s$].

Group	*N*	Tumor resection rate		VAS Scoring (Points)	
		Complete resection	Partial residue	1 day after operation	3 days after operation
Control group	37	34 (91.89)	3 (8.11)	3.54 ± 1.44	2.51 ± 1.13
Observation group	32	30 (93.75)	2 (6.25)	2.81 ± 1.49	1.97 ± 0.88
*χ* ^*2*^ */t*		0.212		2.066	2.189
*P*		0.644		0.043	0.032

**Table 4:** Comparison of complications after surgical treatment (*N*, %).

Group	*N*	Occurrence of complications					Total incidence rate
		Nerve injury	Dysphagia	Difficulty in opening mouth	Massive hemorrhage	Salivary gland fistula	
Control group	37	5 (13.51)	2 (5.41)	3 (8.11)	2 (5.41)	2 (5.41)	14 (37.84)
Observation group	32	2 (6.25)	1 (3.13)	1 (3.13)	1 (3.13)	0 (0.00)	5 (15.63)
*χ* ^*2*^							4.243
*P*							0.039

## Data Availability

The data sets used and analyzed during the current study can be obtained from the corresponding author upon reasonable request.
